# Meta-Analysis of 3D Printing Applications in Traumatic Fractures

**DOI:** 10.3389/fsurg.2021.696391

**Published:** 2021-08-31

**Authors:** Sha Yang, Huapeng Lin, Cong Luo

**Affiliations:** ^1^Department of Orthopaedics, Children's Hospital of Chongqing Medical University, Chongqing, China; ^2^Ministry of Education Key Laboratory of Child Development and Disorders, Chongqing Key Laboratory of Pediatrics, Chongqing Engineering Research Center of Stem Cell Therapy, National Clinical Research Center for Child Health and Disorders, China International Science and Technology Cooperation Base of Child Development and Critical Disorders, Children's Hospital of Chongqing Medical University, Chongqing, China; ^3^Department of Intensive Care Unit, Affiliated Hangzhou First People's Hospital, Zhejiang University School of Medicine, Hangzhou, China

**Keywords:** 3D printing, meta-analysis, trauma, fracture, effect, safety

## Abstract

**Background:** Traumatic fracture is a common orthopaedic disease, and application of 3D printing technology in fracture treatment, which entails utilisation of pre-operative printed anatomic fracture model, is increasingly gaining popularity. However, effectiveness of 3D printing-assisted surgery lacks evidence-based findings to support its application.

**Materials and Methods:** Embase, PubMed and Cochrane Library databases were systematically searched until October, 2020 to identify relevant studies. All randomised controlled trials (RCTs) comparing efficacy of 3D printing-assisted surgery vs. conventional surgery for traumatic fractures were reviewed. RevMan V.5.3 software was used to conduct meta-analysis.

**Results:** A total of 12 RCTs involving 641 patients were included. Pooled findings showed that 3D printing-assisted surgery had shorter operation duration [standardised mean difference (SMD) = −1.52, 95% confidence interval (CI) – 1.70 ~ −1.34, *P* < 0.00001], less intraoperative blood loss (SMD = 1.34, 95% CI 1.74 ~ 0.94, *P* < 0.00001), fewer intraoperative fluoroscopies (SMD = 1.25, 95% CI 1.64 ~ 0.87, *P* < 0.00001), shorter fracture union time (SMD = −0.15, 95% CI −0.25 ~ −0.05, *P* = 0.003), and higher rate of excellent outcomes (OR = 2.40, 95% CI 1.07 ~ 5.37, *P* = 0.03) compared with conventional surgery. No significant differences in complication rates were observed between the two types of surgery (OR = 0.69, 95% CI 0.69 ~ 1.42, *P* = 0.32).

**Conclusions:** Indicators including operation duration, intraoperative blood loss, number of intraoperative fluoroscopies, fracture union time, and rates of excellent outcomes showed that 3D printing-assisted surgery is a superior alternative in treatment of traumatic fractures compared with conventional surgery. Moreover, the current study did not report significant differences in incidence of complications between the two approaches.

**Systematic Review Registration:** CRD42021239507.

## Introduction

Previous studies report that traumatic fractures are leading causes of death and disability worldwide (1). Traumatic fracture is a common orthopaedic disease that consumes immense amounts of medical health resources (2, 3). Previous studies established that most common mechanism for traumatic fractures include low-energy injuries such as slipping, tripping, and falling, as well as traffic accidents (4). Fracture treatment entail reduction and fixation. Although many traumatic fractures require surgical treatment, conservative treatment is considered for some patients with fractures.

In traditional surgical methods, surgeons make surgical plans according to two-dimensional (2D) imaging techniques such as digital radiography (DR), computerised tomography (CT) and magnetic resonance imaging (MRI). However, these techniques cannot show overlaps and complex shapes of bone pieces, leading to insufficient understanding of fractures, which complicates surgical operation. Previous studies have reported that insufficient understanding of fractures may also increase surgical invasiveness in order to sufficiently expose fracture sites during operation to understand the fracture circumstance. This aggravates tissue damage, prolongs operation time and increases intraoperative blood loss (5). Therefore, therapeutic effects of traditional surgery are unsatisfactory.

Continuous improvement of radiological technology in recent years has led to explosive growth in application of 3D printing technology in surgery and plays key roles in clinical treatment of orthopaedic diseases. 3D printing technology is currently widely used in several orthopaedic surgery programs, ranging from complex fracture types to revision arthroplasty, especially in treatment of traumatic fractures, with 3D printing models providing visual and tactile assistance (5). Studies aver that 3D printing model provides more accurate pictures of fractures, whether preoperatively planned or postoperatively reviewed (6, 7). Before surgery, a 3D printed model allows surgeons to grasp fracture morphology and the relative position of fracture fragments, offer opportunities to set up a complete preoperative plan, such as selection of best operative approach, need for bone grafts, size of the fixture, placement of the fixture and trajectories of screws. Fractures are presented to patients and their families using 3D printed models to facilitate communication with doctors to understand their conditions better and cooperate better during treatment. Furthermore, surgeons can communicate better with work teams, which improves collaboration and performance of working team (7–11). In addition, shape and size of plate can be determined by attaching plate to life-size and accurate 3D fracture model (personalised 1:1 solid fracture prototype). Screws with ideal length, location and orientation of fractures can be selected by placing them on personalised 1:1 solid fracture model. Doctor can then simulate reduction and internal fixation based on 3D model, decide on the best way to fix fracture fragment, and establish complete pre-operative plan.

Recent studies have reported that 3D printing-assisted surgery is more effective compared with traditional surgery in treating all types of fractures. However, these reports are not evidence-based. The current study, explored application of 3D-printing- assisted surgery as a preoperative printed anatomic fracture model in treatment of traumatic fractures.

## Materials and Methods

This study was conducted in accordance with Preferred Reporting Items for Systematic Reviews and Meta-Analyses (PRISMA) guidelines (12) and Cochrane Handbook for Systematic Reviews of Interventions (V.5.0.2).

### Literature Retrieval

The current study searched PubMed, Embase, and Cochrane Library databases from inception to October, 2020. Literature was searched using combinations of text words and MeSH words, including 3D or computer-assisted or rapid prototyping, printing or printer, trauma, fracture, management or treatment and fixation or steel plate, as well as their synonymy and near-synonymy. In addition, references of relevant studies were reviewed. Authors were contacted via e-mail if additional information and necessary data were needed.

### Inclusion and Exclusion Criteria

Inclusion criteria used in the current study included: (1) randomised controlled trials (RCTs); (2) research for traumatic fractures of limbs and pelvis, regardless of exact cause of injury; (3) 3D fracture models were used for preoperative plan to determine where it best secured fracture fragments, suitable metal plates and screws with ideal location, length and orientation; (4) comparing efficacy of 3D-printed assisted surgery with conventional surgery, without 3D printing model, for traumatic fractures; (5) human studies; (6) outcome indicators included operation time, intraoperative blood loss, fluoroscopy times, fracture healing time, anatomic reduction rate. excellent and good rate, as well as complication rate or length of hospital stay.

Exclusion criteria included: (1) research with insufficient data; (2) studies on other types of fractures; (3) non-English articles; (4) non-randomised controlled trials such as case reports, technical reports, animal studies, *in vitro* studies, reviews, and letters.

### Literature Screening and Data Extraction

After exclusion of duplicate literature, two authors independently screened literature, and in cases of disagreement, consensus was reached through discussion or arbitration by third party. Screening process excluded obviously non-conforming literature by reading titles and then further reading abstracts to screen for literature that may be included. After initial screening, full texts were obtained and read to determine whether to include articles. Two authors independently extracted data from included literature according to pre-set data extraction table and reached consensus through discussion or arbitration by third party in cases of disagreement. Extracted information included first name of author, publication year, country, sample size, sex, operative time, intraoperative blood loss, intraoperative numbers of fluoroscopies, fracture union time, excellent and good rates, anatomic reduction rates, complication rates, and length of hospital stay.

### Risk of Bias Assessment

Risk of bias was assessed using criteria outlined by Cochrane back review group (13). Independent evaluation and cross-verification were conducted by two authors. In cases of disagreement, agreement was reached through discussion or arbitration by third party.

### Statistical Analysis

Collected data were statistically analysed using RevMan 5.3 statistical software. For continuous variables, mean differences (MD) were computed as point estimates and their 95% confidence intervals. For different measuring units and large mean differences, SMD was computed. Odds ratio (OR) and 95% confidence interval were computed for dichotomous variables. Heterogeneity of each study (14) was analysed using chi-square test (inspection level for α = 0.1), and *I*^2^-value was used to quantify heterogeneity. *P* < 0.1 or *I*^2^ > 50%, indicated significant heterogeneity among included studies. Reasons for heterogeneity were analysed using subgroup and sensitivity analyses. Random effects model was used for clinically consistent heterogeneity, whereas fixed effects model was used for data without significant heterogeneity. Test level for meta-analysis was set as α = 0.05. Mantel-Haenszel method was used for binary result variables. Inverse variance method was used for continuous outcome variables (fixed effects model was specified). Funnel plots (15) were used to assess possibility of publication bias. Reliability of meta-analysis results was verified using sensitivity analysis to test impact of single data set on findings by removing each single study in turn. Subgroup analysis was undertaken by fracture type (limb and trunk fractures) to determine potential differences between 3D-printed assisted surgery and conventional surgery.

## Results

### Search Results

A total of 1,321 studies were searched, and 12 RCTs with 641 patients were finally included after reading abstracts and full texts (16–27). Details of PRISMA flow diagram of study selection are shown in Figure 1.

**Figure 1:** PRISMA flow diagram of study selection.

### Study Characteristics and Quality Assessment

Types of fractures covered in the current study included pelvic fractures, humeral intercondylar fractures, elbow fractures, proximal humeral fractures, humeral shaft fractures, intra-articular distal radial fractures, femoral intertrochanteric fractures, tibial plateau fractures, trimalleolar fractures, and calcaneal fractures. Operative time was assessed in all included trials, whereas blood loss during surgery was compared in 11 trials and intraoperative X-ray frequency was compared in 7 trials. Moreover, fracture healing time was evaluated in 4 trials, whereas excellent and good rates as well as anatomic reduction rates were each computed in 4 trials. Complications were recorded in 3 trials. Basic features of these studies are shown in Table 1. The studies had been published in the last 5 years and included 641 patients. Bias risk assessment of RCTs is shown in Figure 2. Seven studies that explicitly reported using random sequences for patient group assignment were considered to be of high quality, whereas the other five were of medium quality.

**Table 1:** Basic characteristics of all the RCTs included in this meta-analysis.

**References**	**Country**	**Fracture type**	**Sample (*n*, 3D/C)**	**Gender** **(M/F)**	**Follow-up (month, mean)**	**Time from injury to operation (days, 3D/C)**	**3D fracture model**	**Fixator (3D/C)**	**Outcomes**
Chen et al. (16)	China	Die-Punch fractures	55/52	65/42	13.075	3.19 ± 1.70/ 3.15 ± 1.55	Fracture model: Using CT scan [Star PACS system (INFINITT, Seoul, South Korea)], 3D image was created in Mimics software v10.01 (Materialise, Leuven Belgium); 3D printer (3D ORTHO; Waston Med Inc., Changzhou, Jiangsu, China)	Steel plates and screws, K-wires	Operation time, intraoperative blood loss, number of fluoroscopies
Chen et al. (17)	China	AO type C fractures	23/25	31/17	13.0	3.3 ± 1.8/ 3.7 ± 1.6	Fracture model: Using CT scan [Star PACS system (INFINITT, Seoul, South Korea)], 3D image was created in Mimics software (version 10.01; Materialise, Leuven, Belgium); 3D printer (3D ORTHO; Waston Med Inc., Changzhou, Jiangsu, China)	Metal plates and screws, K-wire	Operation time, intraoperative blood loss, number of fluoroscopies
Shuang et al. (18)	China	Intercondylar humeral fractures	6/7	10/3	10.6	NR	Fracture model: Using CT scan (1 mm), 3D image was created in Mimics v.11.1 software (Materialise, Ann Arbour, MI); 3D printer (SRP400B, Huasen 3D Printing Research, Changzhou, China)	Steel plate and screws, K-wire	Operation time
Maini et al. (19)	India	Acetabulum fracture	10/11	18/3	10.6	≤ 21	Fracture model: Using CT scan, 3D image was created in MIMICS 8.13 software (Materialise, Leuven, Belgium): 3D printing machine EOSINT P380 (EOS, Birmingham, UK) and patient-specific 3D real model was generated using rapid prototyping technology.	3.5 mm reconstruction stainless steel plate	Operation time, intraoperative blood loss
Maini et al. (20)	India	Acetabulum fracture	12/13	23/2	NA	≤ 21	Fracture model: Using CT scan (1 mm), 3D image was created in Mimics software; 3D printer [rapid prototyping technology in poly-lactic acid (PLA)]	Pre-contoured reconstruction plates	Operation time
Kong et al. (21)	China	Intra-articular distal radius fractures	16/16	19/13	6.0	≤ 7	Fracture model: Using CT scan (1 mm), 3D image was created in Mimisc18.0 (Materialise, Belgium) software; 3D printer	K-wire, screws	Operation time, intraoperative blood loss, number of fluoroscopies
Yang et al. (22)	China	Trimalleolar fracture	15/15	16/14	NA	5.4 (4–12)	Model: Using CT scan (1 mm), 3D image was created in Mimics l0.01 software; 3D printer (FlashForge Ltd., ZhengJiang, China). Polylactic acid (PLA) was used as the printing material (FlashForge Ltd., 1.75 mm in diameter)	The internal fixation plate	Operation time, intraoperative blood loss
Yang et al. (23)	China	Elbow fractures	20/20	28/12	10.6	NR	Model: Using CT scan (1 mm), 3D image was created in Mimics 10.01 software; 3D printer (FlashForge Ltd., ZhengJiang, China). PLA and ABS were used as the printing materials (FlashForge Ltd., 1.75 mm in diameter)	Steel plates and screws	Operation time, intraoperative blood loss
You et al. (24)	China	Complex proximal humeral fractures	34/32	39/27	22.3	NR	Model: Using CT scan (1 mm, SIEMENS, Germany), 3D image was created in Mimics 16.0 (Materialise, Belgium); 3D printer [rapid prototyping equipment (3D System Project 660 Pro)]	Steel plates and screws	Operation time, intraoperative blood loss, number of fluoroscopies
Zheng et al. (25)	China	Humeral intercondylar fractures	43/48	49/42	15.5	4.3 ± 1.4 4.2 ± 1.1	Model: Using CT scan [Star PACS system (INFINITT, Seoul, South Korea)], 3D image was created in 3D image was created in Mimics software v15.0 (Materialise, Leuven, Belgium); 3D printer (3D ORTHO Waston Med Inc. Changzhou, Jiangsu, China)	Steel plate and screws	Operation time, intraoperative blood loss, number of fluoroscopies
Zheng et al. (26)	China	Calcaneal Fractures	35/40	44/31	14.8	7.69 ± 2.3/ 7.60 ± 1.7	Model: Using CT scan, 3D image was created in 3D image was created in Mimics software v17.0 (Materialise, Leuven, Belgium); 3D printer (3D ORTHO Waston Med Inc. Changzhou, Jiangsu, China)	Steel plate and screws	Operation time, intraoperative blood loss, number of fluoroscopies
Zheng et al. (27)	China	Pilon fracture	45/48	66/27	20.2	7.6 ± 2.5/ 8.1 ± 2.3	Model: Using CT scan (tar PACS system [INFINITT, Seoul, South Korea)], 3D image was created in Mimics software v17.0 (Materialise, Leuven, Belgium); 3D printer (3D ORTHO Waston Med, Inc., Changzhou, Jiangsu, China)	Metal plates and screws	Operation time, intraoperative blood loss, number of fluoroscopies

**Figure 2:** Risk of bias assessment table and risk of bias assessment chart of RCTs.

### Operation Time

In all included studies (16–27), a total of 641 patients had their operation times reported. Fixed effects model was adopted due to low heterogeneity (*I*^2^ = 43%, *P* = 0.05). Findings showed that operation time for 3D printing-assisted surgery was significantly shorter compared with that for conventional surgery, and pooled SMD was −1.52 (95% CI −1.70 ~ −1.34, *P* < 0.001; Figure 3). Funnel plot did not show any obvious asymmetry (Figure 4).

**Figure 3:** Meta-analysis results of operation time.

**Figure 4:** Funnel plot of included studies.

The included studies were grouped into limb fracture and pelvic fracture groups for subgroup analysis. Data from limb fracture group showed SMD of −1.62 (95% CI −1.80 ~ −1.43, *P* < 0.001) with no significant heterogeneity (*I*^2^ = 0%, *P* = 0.71), whereas data from pelvic fracture group showed SMD of −0.52 (95% CI−1.11 ~ 0.08, *p* = 0.09) with mild heterogeneity (*I*^2^ = 15%, *P* = 0.28).

### Intraoperative Blood Loss

Eleven of the included studies (16, 17, 19–27) reported blood loss in a total of 582 patients. Random effects model was adopted due to significant heterogeneity (*I*^2^ = 78%, *P* < 0.001). Findings showed that intraoperative blood loss in 3D printing-assisted surgery was significantly less compared with that in conventional surgery, and pooled SMD was −1.34 (95% CI −1.74 ~ −0.94, *P* < 0.001; Figure 5).

**Figure 5:** Meta-analysis results of intraoperative blood loss.

Eleven studies were grouped into limb fracture and pelvic fracture groups for subgroup analysis. Findings from limb fracture group showed SMD of −1.53 (95% CI −1.91 ~ −1.16, *P* < 0.001) with significant heterogeneity (*I*^2^ = 74%, *P* < 0.001), whereas findings from pelvic fracture group showed SMD of −0.31 (95% CI −0.89 ~ 0.27, *P* = 0.30) with no heterogeneity (*I*^2^ = 0%, *P* = 0.94).

### Number of Fluoroscopies During the Operation

Seven of the included studies (16, 17, 21, 24–27) reported number of fluoroscopies for a total of 512 patients with limb fractures. Random effects model was adopted due to significant heterogeneity (*I*^2^ = 74%, *P* < 0.001). Findings showed that the number of fluoroscopies in 3D printing-assisted surgery was significantly lower compared with that in conventional surgery, and pooled SMD was −1.25 (95% CI −1.64 ~ −0.87, *P* < 0.001; Figure 6).

**Figure 6:** Meta-analysis results of number of fluoroscopies.

### Fracture Union Time

Four of the included studies (24–27) reported fracture union time for a total of 315 patients with limb fractures. Fixed effects model was adopted due to lack of heterogeneity (*I*^2^ = 0%, *P* = 0.74). Findings showed that fracture union time in 3D printing-assisted surgery was significantly shorter compared with that in conventional surgery, and pooled SMD was −0.15 (95% CI −0.25 ~ −0.05, *P* = 0.003; Figure 7).

**Figure 7:** Meta-analysis results of fracture union time.

### The Rate of Excellent Outcomes

Four studies (18, 19, 26, 27) showed findings on rate of excellent outcomes, where significant differences were observed between 3D printing-assisted surgery and conventional surgery groups (OR = 2.40, 95% CI 1.07 ~ 5.37, *p* = 0.03; *I*^2^ = 0%, *p* = 0.72; Figure 8).

**Figure 8:** Meta-analysis results of the rate of excellent outcomes.

### Complication Rates

Three studies (23, 26, 27) showed data on complication rates. Findings of the current study showed no significant differences in complication rates between 3D printing-assisted surgery and conventional surgery groups (OR = 0.69, 95% CI 0.69 ~ 1.42, *P* = 0.32; *I*^2^ = 0%, *P* = 0.85; Figure 9).

**Figure 9:** Meta-analysis results of complication rate.

## Discussion

Previous studies have report that incidence of traumatic fractures has increased in recent years, which increases consumption of scarce medical resources and adversely affects quality of life of patients, leading to disability and death (28–31). Most traumatic fractures require surgical treatment to fix broken bone and restore its length and anatomic position for faster and full function (32). In traditional surgery, orthopaedic surgeons make surgical plans mainly based on 2D radiographic images. However, 2D images do not accurately show traumatic fractures, especially comminuted fractures.

Rapid development of 3D printing technology has led to its increasing application in orthopaedics (33–42). Type and complexity of fractures vary from person to person. Design of traditional orthopaedic surgery is based more on clinical experience of the surgeon due to inaccuracy of 2D images in showing fractures. However, 3D printing technology creates personalised, accurate, and solid model of fractures (43). 3D-printed model helps orthopaedic doctors develop personalised, accurate and reasonable surgical plans for patients and increase success rates of surgery (44, 45). Previous studies aver that primary surgeons can observe anatomical structures of fractures through 3D-printed prototypes prior to implementation of complicated fracture surgery (46–48) to simulate surgical operation and determine bone block. This is undertaken by simulating screw implantation according to location of patient and direction of internal fixation apparatus, which greatly improves accuracy and safety of screw implantation. Prototype helps to reduce complexity of operation and shorten learning curve (49, 50). 3D printing technology, therefore, helps in clinical diagnosis, in planning complex surgical strategies, simulate surgery, reduce intraoperative injuries, and render diagnosis and surgical operation more intuitive, realistic and specific (51–58). In addition, previous studies report that 3D modelling reduces risk of radiation exposure to patients and surgeons (59).

Previous studies aver that besides improving surgery, doctor-patient communication is also an important part of treatment (60). 3D-printed models have been reported to improve patient understanding and compliance during orthopaedic surgery. Patients and their families are satisfied with this communication method, which effectively improves ability of patients or their families to understand condition of the patients and improves patients' attitude and compliance with doctors' advice, thereby reducing risk of medical disputes (61). Previous studies have established that when 3D fracture model is introduced to help explain condition and operation plan to patients and their families, overall evaluation of quality of doctor-patient communication by patients is above 9 points (27). Besides helping doctors better communicate with patients, use of 3D fracture model improves communication among surgical team members, which increases patients' understanding and compliance and improves performance as well as cooperation ability of surgical team. Furthermore, it can be used in medical teaching to improve understanding (62).

The current meta-analysis established that 3D printing-assisted surgery has great advantages over traditional surgery in terms of operation time, intraoperative blood loss, number of fluoroscopies, fracture union time, rate of excellent outcomes, and anatomical reduction. Moreover, there were no significant differences in complication rates between the two studied groups. However, high heterogeneity among studies cannot be ignored, which may be related to professional skills of surgeons, position and complexity of fractures as well as accuracy of instruments and equipment. More RCTs are needed in future to analyse each fracture type individually to reach more reliable conclusions.

A previous study by Lou et al. (63) was excluded in the current study because the reported SD of operation time and intraoperative blood loss were unbelievably too small to achieve in an actual operation, which would have caused extreme heterogeneity. Sensitivity analysis indicated that each included study did not drive the findings. Trim and fill method indicated that findings of the current study were not affected by publication bias.

However, the current study had some limitations. First, the current study included several different types of fractures, which may have influenced reliability of study findings and may also account for high heterogeneity of findings. Although subgroup analyses were undertaken based on study design, findings may still have been biassed. Second, incidence of type I and type II errors was potentially increased in the current study as raw data were not available. Furthermore, some of the included studies came from the same research group at similar times, which may have led to bias in the findings. Moreover, publication bias was examined only using operation time due to limited number of included studies. Furthermore, only 3 or 4 studies were included for some of outcomes because some studies did not provide data for some results. Finally, sources of high heterogeneity of some results were not analysed in the current study due to insufficient number of included studies.

With rapid development of 3D printing technology, many comparative studies on relative efficacy and convenience of 3D printing-assisted surgery and conventional surgery should be undertaken in future to provide clearer guidance for clinicians to decide on reasonable preoperative plans for traumatic fractures.

## Conclusions

The current study established that 3D printing-assisted surgery has more advantages than traditional surgery in treatment of traumatic fractures. It can, therefore, be included in clinical application. However, multicentre, large samples and well-designed randomised controlled trials are needed to further verify these findings and to study cost-effectiveness of 3D printing for greater benefits to patients.

## Data Availability Statement

The original contributions presented in the study are included in the article/supplementary material, further inquiries can be directed to the corresponding author/s.

## Author Contributions

SY was involved in the conception and design of the study, acquisition of data, analysis and interpretation of data, drafting the article, and final approval of the version to be submitted. HL was involved in the conception and design of the study, acquisition of data, revising the article critically for important intellectual content, and final approval of the version to be submitted. CL was involved in the conception and design of the study, analysis and interpretation of data, revising the article critically for important intellectual content, and final approval of the version to be submitted. All authors contributed to the article and approved the submitted version.

## Conflict of Interest

The authors declare that the research was conducted in the absence of any commercial or financial relationships that could be construed as a potential conflict of interest.

## Publisher's Note

All claims expressed in this article are solely those of the authors and do not necessarily represent those of their affiliated organizations, or those of the publisher, the editors and the reviewers. Any product that may be evaluated in this article, or claim that may be made by its manufacturer, is not guaranteed or endorsed by the publisher.
